The article "Construction of Tourism E-Commerce Platform Based on Artificial Intelligence Algorithm" was retracted in 2023. Reasons: suspected computer-generated content; unreliable results or conclusions; concerns about the data; concerns about the results or conclusions.

# Construction of Tourism E-Commerce Platform Based on Artificial Intelligence Algorithm

**DOI:** 10.1155/2022/5558011

**Published:** 2022-06-10

**Authors:** Xiaoyin Yin, Jiangnan He

**Affiliations:** ^1^Lancang-Mekong International Vocational Institute, Yunnan Minzu University, Kunming 650000, Yunnan, China; ^2^Business School, Yunnan University of Finance and Economics, Kunming 650221, Yunnan, China

## Abstract

In the late twentieth century, with the rapid development of the Internet, e-commerce has emerged rapidly, which has changed the way people travel around the world. The greatest advantages of e-commerce are the flow of information and data and the importance of traveling freely to experience the mind and body in different fields. Tourism is an important part of the development of e-commerce, but the development of e-commerce tourism lags behind. To solve the current situation of the backward development of tourism e-commerce, this article studies the construction of a tourism e-commerce platform based on an artificial intelligence algorithm. By introducing modern information technology, based on a cloud computing platform, big data analysis, K-means, and other key technologies, this article solves the current situation of the development of an e-commerce platform. It also analyzes the construction methods of traditional cloud platforms and modern cloud platforms through comparative analysis and solves the construction methods suitable for artificial intelligence tourism. At the same time, combined with the actual situation of tourism, this article selects the appropriate networking method based on the analysis of the advantages and disadvantages of wired and wireless coverage methods and economics to complete the project design. Its purpose is to ensure that the work meets the specific construction needs and build an artificial intelligence-based smart tourism big data analysis model. It promotes the development of tourism e-commerce industry. It saves costs and improves efficiency for travel service providers. Then, according to the actual situation of tourism, it conducts demand analysis from the perspectives of tourists, scenic spots, service providers, tourism administrative agencies, etc. Experiments show that, through the practical application of the artificial intelligence tourism mobile e-commerce platform in this article, it can be seen that the artificial intelligence tourism mobile e-commerce platform designed in this article can meet the needs of customers for shopping-related tourism commodities. Tourists of attractions have increased by 3.54%, and the economy of tourist destinations has increased by 4.2%.

## 1. Introduction

With the rapid development of economic and social systems, people spend more time and energy to improve the quality of life, which accelerates the development of the current labor market. As one of the most important contents of the service industry, tourism is an important part of project development. The development of tourism services and e-commerce platforms has played an important role in the rapid growth of tourism and the growth of GDP. Due to the slow development of e-commerce travel platforms, it may not be able to meet the different needs of travelers. In this article, the construction of smart travel service can accurately analyze the needs of travelers through e-commerce. The improvement in customer satisfaction is of great significance to the growth of GDP in the tourism industry.

E-commerce business refers to a networked business system as the main body, using the most advanced electronic system for the operation of travel agencies, travel information release systems, and transaction banks based on electronic databases. There are many teams working on it. Fararni, Nafis, and Aghoutane conducted an in-depth exploration of user interaction and information search. They analyzed and concluded that the research on tourism intelligent system will make great contributions to tourism consumption, tourism experience, and tourism workflow [1]. Kotiloglu provides users with accurate personal travel information services through intelligent terminal analysis [2]. Avoliot and Gardner put forward the research on the understanding and management of service supply chain, which has opened up a precedent for the research of service industry supply chain [3]. Kim, Kandampully, and Bilgihan mentioned the planning and concept of smart tourism in “Smart Tourism Analysis.” It starts from the market and builds a central management platform and a traffic information management system. It also builds smart hotels and smart scenic spots [4]. He, Huang, and Huang started from the composition, value, and development trend of smart tourism and pointed out that smart tourism will lead the tourism industry [5]. GuoY, WangM, and LiX, combined with the current situation of e-commerce tourism platform construction, analyzed the problems existing in the construction of e-commerce tourism platform and put forward relevant analysis and suggestions [6]. Huang, Chai, and Yi analyzed the use of e-commerce industry on mobile devices. He analyzed the development status of mobile e-commerce platforms, which provided guidance for the in-depth development of mobile e-commerce [7].

With the development of network technology, the field of artificial intelligence algorithm application has become increasingly extensive, and many teams are currently conducting related research on it. Hou et al. used a combination of artificial intelligence and traditional simulation platforms to build an intelligent self-game platform. The results of their 1V1 air combat simulation experiments show that it has reference significance for promoting the future intelligence of military simulation [8]. Yang S's artificial intelligence-based IoT platform built and analyzed artificial intelligence technology. He studied the development status and trends of artificial intelligence in IoT platforms and discussed the technologies and applications of various AI IoT platforms [9]. Based on the exploration of electronic engineering under artificial intelligence, Yun-he introduced artificial intelligence technology and electronic engineering, aiming to provide a reference for related research and practice [10]. Juszczyk Micha studied the development of artificial intelligence technology to estimate the cost of construction projects. It further elaborates the cost estimation of construction projects based on artificial intelligence technology [11]. CriadoJI Gil-GarciaJR introduced the concept of artificial intelligence. They studied the effective strategies and development trends brought by artificial intelligence technology to the network education platform [12]. Fazekas Ferencfazekas investigated the development history, status quo, and relationship with knowledge services of artificial intelligence to build a knowledge service system model based on artificial intelligence from the perspective of intellectual movable property value promotion chain [13]. Based on the new development background of artificial intelligence technology, Qin J, Li H, and Chen X constructed an information fusion model of intelligent information technology and open education nontechnical support services by combining the characteristics of open education nonacademic support services [14].

This article uses artificial intelligence, service platform construction, recommendation algorithm, and big data mining and other technologies to analyze and construct a tourism database on the basis of understanding the big data cloud platform. It increases customer satisfaction with the e-commerce platform, meets the diverse needs of travel customers, and realizes intelligent travel services.

The innovation of this article:

1. This article adopts artificial intelligence algorithms and K-means and other technologies, which provide strong support for massive tourism information.
2. The platform includes two functions: front-end display and front-end control system reflecting the characteristics of the portal. The back-end mainly provides the company with effective and accurate end-to-end control.
3. The platform automatically collects customer feedback and accurately pushes relevant information to customers according to their opinions.

## 2. Construction of Tourism E-Commerce Platform

### 2.1. Network Architecture

The artificial intelligence tourism management system not only records the basic information of the attractions, but also records all travel information of the passengers who have purchased tickets. In developing the research model, this article was initially based on a consumer satisfaction index combined with an e-commerce platform. Combined with the characteristics of mobile terminals, this article finally accepts the customer satisfaction model embedded in this article. From the user satisfaction index model, this article emphasizes the importance of observing prices. Observation price is determined by product quality. Therefore, for consumers, the quality of the products they buy is an important factor affecting their satisfaction. Therefore, in the design, this work takes the product quality and the product's relevance to the customer's life as the factors affecting customer satisfaction. The system network architecture is shown in Figure 1.

### 2.2. Tourism Information and Mining Based on Artificial Intelligence Algorithm

The big data travel analysis platform provides data for efficient travel data collection, scale management information, business process analysis, and performance optimization through the extraction, analysis, and processing of relevant big data. It includes the construction of intermediate sources and big data analysis and processing systems.

#### 2.2.1. Resource Aggregation Middleware

The task of resource aggregation middleware is to filter, compile, and sort multiple sources, data sources, and service sources as well as refine and quantify shared sources, enabling complex source collection processes. At the same time, while advancing the project, it also focuses on the development of perception technology and the ability of human performance. It undertakes the function of promoting personal services to end users. The intermediate platform can combine multiple application sources (SaaS), multiple business database data sources, product and data storage sources, and multiple service sources published by the service bus.

#### 2.2.2. Big Data Analysis and Processing System

The big data monitoring platform and monitoring objects are shown in Figure 2: e-commerce platforms with a wide range of customers, a wide range of application services, different data types, and high-quality services are difficult to be accepted by customers relying on a single database. Only by analyzing the needs of customers can we achieve customer satisfaction.

### 2.3. Intelligent Analysis of Tourist Behavior

Statistical analysis of tourists is a typical feature of the current data mining period. Through the analysis and improvement in these data sets, it will play an important role in the travel of tourists.  Figure 3 shows the background control mechanism for travelers' interest preferences.

Through analytics services, it can play an important role in promoting the performance of landscaped sites. It can also provide travelers with information services according to different months, such as local customs, accommodation planning, and meals. From the analysis in Figure 3, it can be seen that managers can analyze the interests and hobbies of tourists. It can analyze individual differences and general analysis of member data, which provides satisfactory service to travelers. The overall analysis and evaluation of tourists can accurately predict tourists' hobbies and shopping needs, thereby driving the development of related industries. At the same time, combined with the comparison of the same period in previous years and horizontal comparison, it can provide data support for all tourist attraction services.

### 2.4. Service System Architecture Based on Tourism E-Commerce

As a system support, the service platform provides services and maintenance of the entire service system through data exchange methods such as connection technology and data entry. Data sources come from business development such as data warehouses, retailers, hotel reservations, etc. Designing personal travel ideas is based on database decisions. This article uses well-known experts and professionals in the travel field as the application model library. This article uses the most common analysis methods, such as short-term analysis. It depends on the traveler's travel time, consumption level, personal needs, etc. It realizes a systematic understanding of travel routes and automatically simulates the best route based on existing data. While combining relevant data, this article considers the impact of virtual travel and makes appropriate changes based on the traveler's results. It finds the right solution for the traveler's personal trip. It also supports the idea of planning personal trips by analyzing customer preferences and behaviors [15] (Figure 4).

In the business model of the e-commerce platform, travel agencies such as scenic spots, hotels, travel agencies, and car rental companies provide services in the e-commerce travel space through standard service interfaces. Travelers can find the travel information they need through e-commerce travel platforms or directly according to their needs. The e-commerce tourism platform provides a display platform for many tourism enterprises, simplifies the transaction process, promotes the horizontal integration of tourism resources, and increases the market vitality and competitiveness of the tourism industry.

At the same time, as an independent third-party trading platform, it has also become an intermediary and bridge between travel service providers and travelers. Travelers can obtain more reliable travel product information through e-commerce travel platforms. It involves many small and medium-sized travel companies, and travelers have more choices and opportunities in comparison to travel use. The role of building a tourism e-commerce platform to promote tourism development is as follows:

#### 2.4.1. Promotes Resource Integration and Provides Multilevel Services

One is to promote the horizontal integration of tourist sources. Due to the low level of informatization of travel agencies, most travel agency websites only provide simple information to some small and medium-sized travel agencies, hotels, and other browsers. It does not have its own website, attractions, hotels, luggage, and facilities. Other itineraries are generally coordinated by the travel agency's itinerary, which hinders the large-scale cooperation between travel agencies and the integration of travel sources. With the introduction of standard SOA services, the e-commerce platform is connected with the distributed information systems of multiple travel companies. It ensures the real time and completeness of the products and travel services provided by the e-commerce platform. As an independent third-party transaction platform, the travel e-commerce platform provides travel agencies, especially small travel agencies, hotels, and freighters, with information and transactions to promote products and services and provide platforms. It provides credit guarantees for their products and services. It has conquered more product worlds for small and medium travel companies. It provides travelers with more levels of products and travel services.

#### 2.4.2. Saves Economy and Resources and Realizes Cross-Platform Cooperation

Second, it saves travel companies' financial and human resources due to the lack of a good way to connect many companies' information systems. This makes it difficult for top suppliers to actually build an online network. The first reason is that platform integration needs to rely on different Internet environments, in which case a custom integration scheme is not enough. The easy integration of AI algorithms creates favorable conditions for the B2B2C model. First, end-to-end integrated systems allow companies to reuse existing IT capabilities to create e-commerce business plans. E-commerce is not a competitive technology for existing large travel companies and large travel exchange platforms and does not require reinventing new applications. Second, the simple integration provides a multi-channel approach that makes it possible to simplify communication between very disparate systems in the current e-commerce travel space. The e-commerce platform allows AI algorithms to connect to different travel information systems and services of many travel companies through standard service interfaces. The information is provided in real time on the e-commerce travel platform, which does not require a lot of investment and improvements on existing software and applications, saving the economy and resources of the company's human resources.

#### 2.4.3. Provides Reliable Real-Time Information to Meet the Individual Needs of Passengers

Finally, it provides travelers (especially foreign travelers) with complete and reliable real-time information on tourism products and services, but people still know little about the customs and habits of tourist destinations. The e-commerce travel platform provides credit insurance for the products and services of all participating travel companies, allowing travelers to choose travel products and related services with confidence. It can also choose individual tours, such as personal needs and hobbies. It can also invite other ALICE friends to travel together in the ALICE area [16].

### 2.5. E-Commerce Platform Ticketing Order System

Vision electronic ticketing plan: The first is to provide ticketing services for tourist attractions. The second is to provide online ticketing services for affiliated companies through the Internet and network platforms. The on-site ticketing system can meet the regulatory framework of product promotion services, financial services, and guidance services by focusing on a wide range of resources. The e-ticket system is shown in Figure 5.

In this article, the electronic ticketing system is used to replace the rough and disorderly management method with the control of refinement, control, and adjustment at any time. It is not only convenient for travelers, but also reduces the cost of landscape control and production.

### 2.6. Artificial Intelligence Algorithm

The artificial intelligence algorithm includes two parts [17], namely the forward propagation of the signal and the back propagation of the error. The application of this structure has established that individuals can use algorithmic signal propagation in both directions for regular training to achieve the accuracy of predicted outcomes.

In this article, *n*, *l*, *m* are used to denote the number of entry points, hidden nodes, and output nodes in the network, respectively. It uses, *Q*_(*iji*=1,2,…,*n*; *j*=1,2 …,*l*,)_ to represent the weight between the input node and the hidden node, and *Q*_*jk*_(*j*=1,2,…, *l*, *k*=1,2,…*m*) to represent the relationship between the hidden nodes. The neurons of the hidden node and the output node are selected as the sigmoidal function, and the output node and the weights are as follows:

(1) $$\begin{array}{c} f\left(x\right)=\frac{1}{1+e^{-\gamma x}}. \end{array}$$

Let *K* represent the input value of training data, *K*={*k*_1,_k_2Ω_,…, *k*_*n*_}, and use *P* to represent the expected output, *P*={*p*_1,_*p*_2_,…, *p*_*n*_}, so that all artificial intelligence input general terms can be determined, namely

(2) $$\begin{array}{c} H_{j}=\overset{n}{\underset{i=1}{Μ}}\omega_{ij}x_{i}i,=1,2,\ldots ,n,\text{d}=1,2,\ldots ,l. \end{array}$$

To reduce the difficulty of calculation work, in general, we will assume *λ*=1, and then we can determine the output results of different hidden nodes:

(3) $$\begin{array}{c} {\text{net}}_{l}=f\left(H_{j}\right)k=1,2,\ldots ,l. \end{array}$$

The input to the output node is

(4) $$\begin{array}{c} O_{k}=\sum_{j=1}^{1}H_{j}\omega_{jk}k=1,2,\ldots ,n. \end{array}$$

Possible output results are

(5) $$\begin{array}{c} y_{i}=f\left(O_{k}\right)q=1,2,\ldots ,m. \end{array}$$

Using *d*_1_ to represent the magnitude of the output BP network nervous system numbered, then the prediction error of the neuron is

(6) $$\begin{array}{c} e_{i}={\text{d}}_{1}-y_{1}. \end{array}$$

From this, the function for calculating the error of the output layer can be determined as follows:

(7) $$\begin{array}{c} B=\frac{1}{2}\sum_{i}e_{i}^{2}\\ =\frac{1}{2}{\left(d_{i}-y_{i}\right)}^{2}. \end{array}$$

Then, the error data transfer formula between the input layer and the hidden layer is

(8) $$\begin{array}{c} \Delta \omega_{ij}=-\eta \frac{\alpha E}{\alpha \omega_{ij}}i=1,2,\ldots ,n,j=1,2,\ldots ,m.s. \end{array}$$

The error transfer data formula between the output layer and the hidden layer is

(9) $$\begin{array}{c} \Delta \Phi_{jk}=-\eta \frac{\partial E}{\partial \omega_{jk}}j=1,2,\ldots ,g,k=1,2,\ldots ,m. \end{array}$$

Among them

(10) $$\begin{array}{c} \frac{\partial G}{\partial \omega_{jk}}=\frac{\partial E}{\partial y_{i}}\frac{\partial y_{j}}{\partial \omega_{jk}},\\ \frac{\partial E}{\partial y_{i}}=-\left({\text{d}}_{1}-y_{1}\right),\\ \frac{\partial y_{i}}{\partial y_{1}}=\frac{\partial y_{1}}{\partial O_{i}}\frac{\partial O_{i}}{\partial \omega_{jk}}. \end{array}$$

Because artificial intelligence nonlinear excitation Sigmoid function satisfies the following relation:

(11) $$\begin{array}{c} f\prime \left(a\right)=f\left(a\right)\left(1-f\left(a\right)\right). \end{array}$$

After combining (3), (12), and (13), we get

(12) $$\begin{array}{c} \frac{\partial y_{1}}{\partial \omega_{jk}}=y_{1}\left(1-y_{1}\right){\text{net}}_{j}. \end{array}$$

At this point, the result of formula (9) is calculated as follows:

(13) $$\begin{array}{c} \Delta \omega_{jk}=-\mu \left({\text{d}}_{i}-y_{i}\right)y_{i}\left(1-y_{i}\right){\text{net}}_{j}. \end{array}$$

In addition, there are

(14) $$\begin{array}{c} \frac{\partial {\text{y}}_{k}}{\partial {\text{net}}_{j}}=\frac{\partial y_{k}}{\partial O_{k}}\frac{\partial O_{k}}{\partial {\text{net}}_{j}},\\ =y_{k}\left(1-y_{k}\right)\omega_{ki},\\ \frac{\partial {\text{net}}_{j}}{\partial \omega_{ij}}=\frac{\partial {\text{net}}_{j}}{\partial H_{i}}\frac{\partial H_{i}}{\partial \omega_{ij}},\\ ={\text{net}}_{j}\left(1-{\text{net}}_{j}\right)\kappa_{j}. \end{array}$$

Converting formula (15) into the following form:

(15) $$\begin{array}{c} \Delta \omega_{jk}=-\eta \sum_{k=1}^{m}\left({\text{d}}_{k}-y_{k}\right)y_{k}\left(l-y_{k}\right){\text{net}}_{i}\left(1-{\text{net}}_{i}\right)x_{j}. \end{array}$$

Then according to formulas (1) to (16), the general formula for calculating the relationship between the input layer and the hidden layer, and the hidden layer and the output layer in the neural network is as follows:

(16) $$\begin{array}{c} \omega_{ij}\left(t+1\right)=\omega \left(t\right)+\Delta \omega_{jk},\\ =p\overset{m}{\underset{k=1}{\sum }}\left({\text{d}}_{k}-y_{k}\right)y_{k}\left(l-y_{k}\right){\text{net}}_{i}\left(1-{\text{net}}_{i}\right)x_{j},\\ i=1,2,\ldots ,n,j=1,2,\ldots ,m,\\ \omega_{jk}\left(\left(t+1\right)=\omega_{jk}\left(t\right)+\sum \left({\text{d}}_{i}-y_{i}\right)y_{i}\left(1-y_{i}\right)\right){\text{net}}_{j},\\ i=1,2,\ldots ,n,j=1,2,\ldots ,l,k=1,2,\ldots ,m. \end{array}$$

The above process is a training step of the artificial intelligence network [18, 19]. Given that the algorithmic error is the nature of backward evolution, during the execution of the training step, the density of each layer is continuously adjusted to keep the error to a minimum [6].

The K-mean algorithm is a classical grouping algorithm in nontraining learning. It is based on the basic premise of “gather people and divide people,” and classifies similar parts in unstructured data samples into the same category. The implementation process is as follows: ① Randomly selecting *k* elements as the initial cluster center. ② Calculating the distance from each object to each cluster center, and assigning each object to the nearest cluster center. ③ Recalculating the center of the cluster, and repeat ② until the end state is satisfied. The termination state can be empty and then assigned to the cluster center, or it can be the quadrature error of the cluster center and the smallest region, etc.

The application field of K-means clustering algorithm is very wide, which can be applied to text recognition and image segmentation. In practice, as long as it is about data clustering application scenarios, it can be used such as map coordinate aggregation, malicious traffic attack identification, etc.

The Apriori algorithm is a very classic algorithm for extracting repetitive applications. For example, FP-Wood, GSP, and CBA are all based on the Apriori algorithm. The process of the Apriori algorithm is as follows: ① Setting up the support portal. ② Examining the entire data set, counting the number of events for each item, and calculating the appropriate support for each item. ③ Clipping out objects below the support threshold and then connecting other objects is a binomial system, that is each object has two elements. ④ Rescanning the entire data set. ⑤ Cutting off the binomial program at the bottom of the support port, and then connecting the other binomial programs into three components, that is each component has three components. ⑥ Repeating ④ and ⑤ until the object set *k* cannot be linked to the object of set *k* + 1. The currently defined object *k* is the data system to be extracted.

The Apriori algorithm is widely used in supermarket shopping data systems, e-commerce shopping data systems, etc., which facilitates the transportation of related products or related store products.

## 3. Experiment of Tourism E-Commerce Platform

To understand the impact of e-commerce tourism on the development of tourism economy, this work takes 2017 as a cross section and selects the annual research project “Tourism Information and E-Commerce Report” of a local e-commerce research company A. It takes the data provided by the annual statistical yearbook issued by the local statistical bureau as a sample, and this article conducts correlation analysis and linear regression analysis model verification (Figure 6).

Among them, the total revenue of tourism companies in a certain region is used as the dependent variable. The number of Internet companies can measure the development level of tourism e-commerce, and the overall level of Internet applications, the scale of platform companies, and the general level of platform applications are used as independent variables.

They are respectively set as *l*_1_, *l*_2_, *l*_3_, and *l*_4_. In this article, the SPSS statistical software is used to analyze the compatibility of the five travel variables, and the results are shown in Figure 7.

The results show that the total tourism revenue *y* is related to the total level of network companies *l*_1_, the number of platform companies *l*_2_, and the number of platform companies *l*_3_, The correlation ratios of *l*_4_ for the total level of platform application were 0.955, 0.963, 0.892, and 0.894, respectively. The correlation coefficients are the test probabilities *P* that are all close to 1. Therefore, the analysis results show that there is a significant positive correlation between the number of websites, the overall level of network applications, the number of platform companies, and the overall level of platform resources and costs. That is to say, the development of e-commerce tourism has had a significant impact on the tourism industry and has a positive effect on the growth of the economy.

To further examine the impact of e-commerce business on the development of the tourism system, the following linear regression analysis method was used to calculate and analyze the four independent variables to determine their specific impact on tourism revenue (Figure 8).

It can be seen from the reflection in the above figure that the overall level of the application of the travel company's website and the overall level of the application of the travel company's e-commerce platform has the greatest impact on the overall income of the tourism industry. These two characteristics also affect the development of the tourism system and play a promoting role.

## 4. Results of Travel E-Commerce Platform

### 4.1. Usage of Tourism E-Commerce Platform in the Context of Artificial Intelligence

This study preliminarily explores customer satisfaction with e-commerce mobile travel platforms. This article also understands the current usage, customer sharing, and specific functions of the mobile e-commerce platform through research (Figure 9).

The results show that through the survey, tourists can use the e-commerce platform to book high-speed rail tickets, hotels, scenic spots, tickets in advance, and view the routes of surrounding scenic spots. The artificial intelligence tourism mobile e-commerce platform designed in this article can meet 90% of customers' shopping needs for tourism commodities.

### 4.2. Tourism Test Based on Paper System

Based on the e-commerce system of artificial intelligence algorithm, this article tests the number of tourists in a famous tourist attraction and also selects several varieties. They are the number of passengers from February to November in 2017, from February to November in 2018, and from February to November in 2019 after introducing artificial intelligence algorithms into the travel e-commerce platform (Figure 10).

The results show that it can be seen from the statistics that the total number of people who introduced artificial intelligence algorithms into e-commerce platforms in 2019 increased by 3.54% year-on-year compared to 2017.

After introducing the artificial intelligence algorithm into the tourism e-commerce platform, the economic growth of a famous tourist attraction was analyzed. This article selects the operating sales of each month in 2017 and 2018 and the monthly sales growth after the introduction of artificial intelligence algorithms in 2019 and 2020 (Figure 11).

The results show that after the introduction of artificial intelligence algorithms into the tourism e-commerce platform, the economy of a tourist attraction has grown by 4.2% annually.

## 5. Discussion

This article summarizes the user operating system of the e-commerce platform. It uses artificial intelligence algorithms to analyze all aspects of platform travel information. It analyzes the individual preferences and needs of different users and designs the entire platform according to the operating system and user requirements, including system architecture, data design, and system design. The design and implementation of the system completes all functions of the system design. The user information management module mainly realizes the input function of user information initialization and real-name authentication information initialization and tests the entire operation process of the travel e-commerce platform and the system load. This article identifies the data entry and conversion of different users according to the test platform. It can understand functions such as store creation, information printing, product purchasing, and reservation services.

## 6. Conclusion

From the perspective of artificial intelligence algorithms, this article deeply discusses the relationship between smart tourism and tourism e-commerce development and the innovation and promotion effect on tourism development. On this basis, this article attempts to propose a smart tourism construction plan and carries out the overall design and detailed implementation design. It makes an in-depth analysis of the operation mechanism, form, technology, and function of realization. Through the discussion and research of the full text, the following conclusions are drawn:

1. This article integrates information into the tourism system, e-commerce tourism has changed many elements of the system: the relationship between the elements, the architecture, the design process, and the relationship between the system and the environment. This process will expand the travel system, making the attributes and services of the travel system change.
2. Information technologies such as artificial intelligence algorithms play an important supporting role in the design of smart travel services. It is also a key driving force for the innovation and construction of smart travel systems. The introduction of modern information technology is not only the recognition of technological innovation in the development of the tourism industry, but also the understanding of the internal organization, innovation, management and control, planning, marketing, and sales of the tourism industry, which realizes the innovation of the entire tourism industry.
3. This article presents the construction of an e-commerce service system based on modern information technology that will introduce new productivity and market power. It promotes the transformation of the tourism industry from extensive operations to fine operations, the excessive development of traditional tourism to modern tourism, and the upgrading of the tourism industry and realizes the joint development of tourism across regions. It has developed tourism into a pillar industry and a more advanced industry of the national economy.

## Figures and Tables

**Figure 1:** Network architecture diagram of tourism e-commerce platform.

**Figure 2:** Data analysis and mining process.

**Figure 3:** Sequence diagram of intelligent analysis of passenger preference.

**Figure 4:** Construction of service platform based on tourism e-commerce.

**Figure 5:** The composition of the electronic ticketing system.

**Figure 6:** Travel information and e-commerce report of company A.

**Figure 7:** Compatibility analysis of five travel variables.

**Figure 8:** Impact on total tourism revenue.

**Figure 9:** Platform usage distribution usage amount.

**Figure 10:** Changes in the number of passengers from 2017 to 2019.

**Figure 11:** Changes in tourism sales turnover.

## Data Availability

The data underlying the results presented in the study are available within the article
